The article "Recommending Crowdfunding Project: A Graph Kernel-Based Link Prediction Method for Extremely Sparse Implicit Feedback" was retracted in 2023. Reasons: signs of a paper mill; suspected computer-generated content; unreliable results or conclusions; concerns about the data.

# Recommending Crowdfunding Project: A Graph Kernel-Based Link Prediction Method for Extremely Sparse Implicit Feedback

**DOI:** 10.1155/2022/5126140

**Published:** 2022-07-19

**Authors:** Pei Yin, Ya Chen, Huan Wang, Hongcheng Gan, Ye Zhou

**Affiliations:** ^1^Business School, University of Shanghai for Science and Technology, Shanghai 200093, China; ^2^Office of Assets and Laboratory Management, Tongji University, Shanghai 200092, China

## Abstract

It is a critical task to provide recommendation on implicit feedback, and one of the biggest challenges is extreme data sparsity. To tackle the problem, a graph kernel-based link prediction method is proposed in this paper for recommending crowdfunding projects combining graph computing with collaborative filtering. First of all, an investor-project bipartite graph is established based on transaction histories. Then, a random walk graph kernel is constructed and computed, and a one-class SVM classifier is built for link prediction based on implicit feedback. At last, top N recommendations are made according to the ranking of investor-project pairs. Comparative experiments are conducted and the results show that the proposed method achieves the best performance on extremely sparse implicit feedback and outperforms baselines. This paper is of help to improve the success rate of crowdfunding by personalized recommendation and is of significance to enrich the research in recommendation systems.

## 1. Introduction

Crowdfunding is a new fundraising method that rapidly developed with the rise of the Internet. As the biggest crowdfunding platform, Kickstarter (https://www.kickstarter.com) raised 4,384,962,222 US dollars for 165,564 successfully funded projects by 16,475,171 users up to now. Besides that, the leading European crowdfunding website Ulule (https://www.ulule.com) has 28,294 successfully funded projects, with more than 2.6 million members worldwide, and raised 143,381,350 euros over the last six years. However, the success rate is rather low, with only 37% on Kickstarter and 65% on Ulule. The factors influencing the success rate may be project creativity, advertising exposure, or project duration. But the biggest reason is that such platforms only provide simple categories and search engine, and it is hard for investors to find the projects that they are interested in [1]. Therefore, recommending crowdfunding projects rises in response to such problem.

The survey shows that data sparsity of most crowdfunding platform reaches 99%, and conventional and classic recommendation methods fail to deal with such extremely sparse data. Moreover, implicit feedback requires different recommending method from rating data [2], since it is infeasible to determine whether unhappened transactions indicate impossible link between an investor and a project or possible link that will happen in the future.

The article "Recommending Crowdfunding Project: A Graph Kernel-Based Link Prediction Method for Extremely Sparse Implicit Feedback" was retracted in 2023. Reasons: signs of a paper mill; suspected computer-generated content; unreliable results or conclusions; concerns about the data.

To deal with sparse implicit feedback, the extant related research works are mainly focused on designing collaborative filtering algorithms, which makes recommendation to a user based on the choices made by similar other users [3–6]. However, traditional collaborative filtering methods suffer from strong dependency of data and lack of expansibility, and they are mainly based on linear modeling using simple and stable inner product of eigenvector of user-item matrix, which is not the best choice for estimating the complex and dynamic relevance of users and items.

Transferring the user-item matrix into a bipartite graph, by treating users and items as nodes and user-item interactions as links, collaborative filtering can be naturally transformed into a link prediction problem in the graph. Then, a graph-based method is applied to compute the global similarity of graphs. Comparing that only users' or items' similarity is computed in collaborative filtering, in the global iteration process of the graph-based method, not only is the relevance of users and items calculated, but also the relevance of users and the relevance of items are computed. Thus, the graph-based method provides the possibility to alleviate the data sparsity issue in collaborative filtering with graph structure modeling [7–9].

Therefore, this paper is motivated to tackle the problem of extremely sparse implicit feedback and proposes a graph kernel-based link prediction method to extract the implicit and potential relations between investors and projects in online crowdfunding platforms. The remainder of this paper is organized as follows: Section 2 reviews the related literature.  Section 3 proposes the graph kernel-based link predication method.  Section 4 set ups experiment using the data of a popular crowdfunding platform.  Section 5 conducts comparative experiments and evaluates the results.  Section 6 concludes our study.

## 2. Literature Review

### 2.1. Crowdfunding Recommendation

The research on crowdfunding recommendation mainly focuses on two aspects. One is that the recommendation system is constructed based on mathematical model. For example, Vineeth et al. [10] proposed a probabilistic recommendation model called CrowdRec, which recommends projects to investors by combining the ongoing state of the project, the individual investor's preferences, and the collective preferences of groups of investors. Song et al. [11] proposed a recommender system based on a structural econometric model to match returning donors with fundraising activities on charitable crowdfunding platforms by maximizing the utility of altruism (the welfare of others) and egoism (self-motivation). Zhang and Zhang [12] proposed a personalized crowdfunding platform recommendation system based on a multiobjective evolutionary algorithm, which leverages the profit and the variety of recommendations with investors' preferences.

The article "Recommending Crowdfunding Project: A Graph Kernel-Based Link Prediction Method for Extremely Sparse Implicit Feedback" was retracted in 2023. Reasons: signs of a paper mill; suspected computer-generated content; unreliable results or conclusions; concerns about the data.

Moreover, other related research works focus on developing crowdfunding recommenders based on machine learning algorithms. For example, Benin and Adriano [13] compared various machine learning algorithms such as gradient boosting tree, Bayesian belief nets collaborative filtering, and latent semantic collaborative filtering for crowdfunding recommendation. Wang and Chen [14] proposed a bipartite graph-based collaborative filtering model, which calculates the global similarity among nodes by personal rank and makes recommendation through collaborative filtering.

### 2.2. Graph-Based Recommendation Algorithms

As matrix can be easily transferred into graphs, the graph-based recommendation algorithms draw increasing interest from scholars [7, 15]. Bipartite graphs are an expansion of network theory, which has attracted more attention in fields such as social network analysis [16]. Bipartite graphs are different from PageRank. PageRank treats network nodes as homogeneous, while the nodes in a bipartite graph are divided into two types: the nodes of different types that have direct connections and the nodes of the same type that have no direct connections [17]. Crowdfunding networks can be considered as bipartite graphs, in which one type of nodes is investors and the other type is crowdfunding projects. The bipartite graph model is able to calculate the distance between nodes by an appropriate algorithm, which can be naturally translated into the similarity between nodes, such as the mean similarity [18]. In recommender systems, some researchers have proposed reducing the complexity of graph model computation with aggregated bipartite graph model, but the recommended accuracy is reduced [19].

With the development of graph neural networks, recent research works have explored neural graph-based recommendation algorithms with strong ability of learning about entities and their relations [20–22]. Some GNN-based recommenders only consider user-item interactions in graph, while others apply GNNs to model knowledge graphs for recommendation [23–25], which take edges as predefined relations between attributes and entities (investors or users) and thus do not consider the relations between attributes. Li et al. [26] and Su et al. [27] leverage GNNs to perform attribute interaction modeling and aggregation as a graph learning procedure.

The article "Recommending Crowdfunding Project: A Graph Kernel-Based Link Prediction Method for Extremely Sparse Implicit Feedback" was retracted in 2023. Reasons: signs of a paper mill; suspected computer-generated content; unreliable results or conclusions; concerns about the data.

### 2.3. Limitations of the Related Graph-Based Recommenders

It is undeniable that GNN-based algorithms achieved relative success in recommendation, especially when combining with collaborative filtering. However, there are two important limitations in such algorithms. One limitation is that, for user and item embeddings, additional complexity is always introduced by the nonlinear feature transformation in GNN which leads to more computing time and storage space and burdens the efficiency in recommendation. The other limitation is that most of the current GNN-based models could only stack very few layers (e.g., 2 layers), which means that, with the increasing of the stacking layers, the smoothing effect could alleviate data sparsity at first but would result in oversmoothing effect with more layers as the higher layer neighbors tend to be indistinguishable for each node. With limited user-item interaction records in the recommendation especially in the scenario of crowdfunding platforms, the problem of oversmoothing would become more severe with high data sparsity, which would neglect each user's uniqueness and degrade the recommendation performance.

## 3. Methodology

### 3.1. The Proposed Approach Framework

Crowdfunding project recommendation is to estimate the probability that investor *i* will back project *p*. Therefore, it is essential to analyze the structure of subtree containing the nearby investors and projects of focal *i* and *p* in the graphical network and utilize it to predict the connection between *i* and *p*.

Since the more similar the topological context of two investor-project pairs is, the more likely that they may share the same relationship within the pairs, this paper proposes a graph-based method focusing on the kernel function computing the similarity between investor-project pairs based on comparison of neighborhood graph structure of the focal pairs. The basic procedure of the proposed graph kernel-based link predication method is illustrated in Figure 1.

1. *Data Collection*. Transactions between investors and projects are obtained from Ulule, a globally well-known crowdfunding platform, through a web crawler.
2. *Bipartite Graph Extraction*. Investor-project graph is established based on transaction histories, and investors' characteristics and projects' features are also extracted.
3. *Graph Kernel Building*. A graph kernel *k*(·, ·) on investor-project pairs is built to compare the similarity of graph structure.
4. *Graph Kernel Computation*. An efficient computation method is chosen to calculate the graph kernel based on the extent research [28], aiming at less runtime and less CPU consumption.
5. *Link Prediction*. A one-class SVM classifier is built to distinguish positive links from negative ones. Furthermore, top *N* recommendations are made according to predicted confidences ranking of investor-project pairs.

The article "Recommending Crowdfunding Project: A Graph Kernel-Based Link Prediction Method for Extremely Sparse Implicit Feedback" was retracted in 2023. Reasons: signs of a paper mill; suspected computer-generated content; unreliable results or conclusions; concerns about the data.

### 3.2. Bipartite Graph Extraction

The dataset of crowdfunding platform contains the interactions between investors and projects. As a result, in order to extract the bipartite graph of investors and projects, firstly the dataset is turned into a *m* × *n* matrix *M*, in which *m* denotes the number of investors and *n* denotes the number of projects, and then the interaction matrix *M*(*M* ∈ *R*^*m*×*n*^) is turned into an expanded adjacent matrix *A*(*A* ∈ *R*^(*m*+*n*)×(*m*+*n*)^), and the value of the expanding part of matrix *A* is set to be 0, where $A=\left[\begin{array}{cc} 0_{m\times m} & M\\ M^{T} & 0_{n\times n} \end{array}\right]$. In this way, the matrix can be easily converted into an undirected graph. At last, matrix *A* is converted into a bipartite graph, in which the nodes denoting investors can only be connected to the nodes denoting projects, and there is no link between any two investors or projects.

As a result, a bipartite graph *G* is defined as a triplet (*I*, *P*, *E*), where *I* denotes investor set, *P* denotes project set, and *E* denotes the links between investors and projects.  Figure 2 shows an example of bipartite graph containing 4 investors (*A*, *B*, *C*, *D*) and 4 projects (*e*, *f*, *g*, *h*), and an edge represents a transaction between an investor and a project.  Figure 3 shows investor-project pairs in the bipartite graph in Figure 2.

As for the features of nodes in the investor-project bipartite graph, all the features are numeric and subtypes and are transformed into one-hot vectors by one-hot coding. The range of values is (0, 1), and the value is 1 only at the *j*-th position and 0 at all other positions.

[000 ⋯ 010 ⋯ 00], *j*-th position.

The value and the processing method of the specific features of investors and projects are shown in Table 1.

### 3.3. Graph Kernel Construction

A kernel function is proposed to quantify the global similarity of graphs; more specifically, the subgraphs contain the neighbors of a focal investor and project pair and predict whether there is a link between the focal investor *i* and project *p* based on the similarity. As a result, the kernel function is given by *K*(*i*, *p*), (*i*′, *p*′).

The similarity of investor-project pairs (*i*, *p*) and (*i*′, *p*′) can be decomposed into the similarity of investors (*i*, *i*′) and the similarity of projects (*p*, *p*′). Thus, the kernel function for comparing the relationships between investors and projects is constructed based on the comparison of entities.

(1) $$\begin{array}{c} K\left(\left(i,p\right),\left(i^{\prime },p^{\prime }\right)\right)=\alpha K\left(i,i^{\prime }\right)+\beta K\left(p,p^{\prime }\right), \end{array}$$

where *α*, *β* ≥ 0 denotes a positive scalar in order to keep it a valid kernel function.

The article "Recommending Crowdfunding Project: A Graph Kernel-Based Link Prediction Method for Extremely Sparse Implicit Feedback" was retracted in 2023. Reasons: signs of a paper mill; suspected computer-generated content; unreliable results or conclusions; concerns about the data.

Random walk is introduced to the kernel function based on a simple idea that performs random walks on a given pair of graphs and counting the number of matching walks. Therefore, paths of random walk on the investor-project graph are generated to capture the semantics inherent in the structure. Moreover, the structure of the investor-project graph is utilized to measure the similarity of investor-project pairs. Given that *G*_*v*_(*v* ∈ {*i*, *i*′, *p*, *p*′}) denotes the subgraphs starting from the focal entities, the kernel function based on random walk can be seen as

(2) $$\begin{array}{c} K\left(\left(i,p\right),\left(i^{\prime },p^{\prime }\right)\right)=\alpha k\left(G_{i},G_{i^{\prime }}^{\prime }\right)+\beta k\left(G_{p},G_{p^{\prime }}^{\prime }\right). \end{array}$$

A random walk path is given as *i*_1_, *i*_2_,…, *i*_t+1_, a transition probability matrix is given as *P*, and the starting probability is given as *p* and the stopping probability is given as *q*. Then a walk's probability is computed as

(3) $$\begin{array}{c} p\left(h|G\right)∶=q_{i_{\left(t+1\right)}}\prod_{j=1}^{\infty }P_{i_{j},i_{\left(j+1\right)}}p_{i_{1}}. \end{array}$$

The random walk graph kernel is defined as the summation of similarities of pairwise paths with the weight of the paths' appearance probability [28].

(4) $$\begin{array}{c} k\left(G,G^{\prime }\right)=\sum_{h}\sum_{h\prime }\sum_{k=1}^{\infty }\mu_{k}k_{\text{path}}\left(h,h^{\prime }\right)P\left(h|G\right)P\left(h^{\prime }|G^{\prime }\right). \end{array}$$

The sequence kernel *k*_path_(*h*, *h*′) represents path similarity of *h* and *h*'. The weight factor *μ*_*k*_ allows the kernel to be flexible by adjusting the value to (de)emphasize walks of different lengths in an application-specific manner.

The similarity of random walk paths center on the focal investor-project pair is computed by decomposing the paths matching into two tasks: nodes matching and links matching [28, 29]. The similarity is set as 0 if the lengths of two paths are different; otherwise, it is calculated as follows:

(5) $$\begin{array}{c} k_{\text{path}}\left(h,h^{\prime }\right)=\prod_{i\in h,i^{\prime }\in h^{\prime }}k_{\text{node}}\left(v_{i},v_{j}^{\prime }\right). \end{array}$$

*k*_node_(·, ·) denotes a node kernel that compares each matching node on the pairwise paths *h* and *h*′.

The article "Recommending Crowdfunding Project: A Graph Kernel-Based Link Prediction Method for Extremely Sparse Implicit Feedback" was retracted in 2023. Reasons: signs of a paper mill; suspected computer-generated content; unreliable results or conclusions; concerns about the data.

The features of nodes are determined by data characteristics and further determine the form of the kernel function; for example, a linear kernel function is more suitable to compute categorical data or textual data [29].

Moreover, the frequently purchased popular products are always listed among the top *N* recommendation, whereas the less popular products are hard to make into the list. Customers of unpopular products are more likely to share common interests than those of popular products. Therefore, it is critical to reduce the effect of products' popularity on node similarity calculation. Based on the idea of TF-IDF, (5) is modified by making proper punishment to popular projects.

(6) $$\begin{array}{c} k_{\text{node}}^{\prime }\left(v_{i},v_{j}^{\prime }\right)=k_{\text{node}}\left(v_{i},v_{\text{node}}^{\prime }\right)\times \frac{1}{\log\left(\left|v_{i}\right|\left|v_{i}^{\prime }\right|\right.}. \end{array}$$

At last, the graph kernel is normalized for more accurate prediction.

(7) $$\begin{array}{c} K^{\prime }\left(\left(i,p\right),\left(i^{\prime },p^{\prime }\right)\right)=\frac{\left.K\left(i,p\right),\left(i^{\prime },p^{\prime }\right)\right)}{\sqrt{\left.K\left(\left(i,p\right),\left(i,p\right)\right)K\left(i^{\prime },p^{\prime }\right),\left(i^{\prime },p^{\prime }\right)\right)}}. \end{array}$$

Equation (7) indicates that the investors or projects farther from the investor-project pair (*i*, *p*) have less influence on predicting the relationship within the pair. Moreover, to deal with the problem of halting [30], a fixed length *k* is utilized and will be optimized by cross validation on the training dataset.

### 3.4. Graph Kernel Computation

The direct product *G*_×_=(*V*_×_, *E*_×_, *φ*_×_) of two graphs *G*=(*V*, *E*, *φ*) and *G*′=(*V*′, *E*′, *φ*′) is defined as follows:

(8) $$\begin{array}{c} V_{\times }=\left\{\left(v,v^{\prime }\right)\in V\times V^{\prime }|\varphi \left(v\right)=\varphi^{\prime }\left(v^{\prime }\right)\right\},\\ E_{\times }=\left\{\left(\left(u,u^{\prime }\right),\left(v,v^{\prime }\right)\right)\in V_{\times }\times V_{\times }^{\prime }|\left(u,v\right)\in E,\left(u^{\prime },v^{\prime }\right)\in E^{\prime },\text{and}\varphi \left(u,v\right)=\varphi {}^{\prime }\left(u^{\prime },v^{\prime }\right)\right\}. \end{array}$$

The runtime complexity of a kernel function based on Kronecker products *O* (*n*^3^) is much more efficient than that of a standard one as *O*(*n*^6^) [31]. Thus, let Kronecker product *G*_×_∶=*G* ⊗ *G*′, adjacency matrix *A*_×_∶=*A* ⊗ *A*′, transition probability matrix *p*_×_ : =*p* ⊗ *p*′, and stopping probability matrix *q*_×_ : =*q* ⊗ *q*′. *A*_×_^*k*^=[vec(*P*)vec(*P*′)^*T*^] represents the probability of random walks with *k* steps on *G*, where the column-stacking operator $\text{vec}\left(P\right)∶=\left[\begin{array}{c} P_{*1}\\ \vdots \\ P_{*m} \end{array}\right]$. Then, the weight matrix *W*_×_ is calculated based on the interaction of Hadamard product and Kronecker product.

(9) $$\begin{array}{c} A_{\times }^{k}☉\left(\hat{\Phi }\left(X\right)⊗\hat{\Phi }\left(X^{\prime }\right)\right)=\left(A^{k}☉\hat{\Phi }\left(X\right)\right)⊗\left(A{{}^{\prime }}^{k}☉\hat{\Phi }\left(X^{\prime }\right)\right)={\tilde{A}}_{\times }^{k}. \end{array}$$

Then, the random walk graph kernel in (5) can be rewritten as follows:

(10) $$\begin{array}{c} k\left(G,G^{\prime }\right)=\sum_{i}^{n}\sum_{i}^{n^{\prime }}\sum_{k=0}^{t}\mu_{k}q_{\times }^{T}{\left[{\tilde{A}}_{\times }^{k}\right]}_{ij}k_{\text{node}}\left(v_{i},v_{i}^{\prime }\right)p_{\times }. \end{array}$$

There are generally four methods developed to compute the random walk graph kernel: Sylvester equations based method, conjugate gradients based method, fixed-point iterations based method, and spectral decompositions based method. The method based on spectral decompositions is chosen in this paper, as it is the most efficient method throughout different application area, but it is only efficient for unlabeled graphs.

The article "Recommending Crowdfunding Project: A Graph Kernel-Based Link Prediction Method for Extremely Sparse Implicit Feedback" was retracted in 2023. Reasons: signs of a paper mill; suspected computer-generated content; unreliable results or conclusions; concerns about the data.

Let ${\tilde{A}}_{\times }^{k}=P_{\times }D_{\times }P_{\times }^{-1}$ denote the spectral decomposition of the graph kernel, in which the columns of *P*_×_ are its eigenvectors and *D*_×_ is a diagonal matrix. Thus, equation (10) can then be rewritten as follows:

(11) $$\begin{array}{c} k\left(G,G^{\prime }\right)=\sum_{i}^{n}\sum_{i}^{n^{\prime }}\sum_{k=0}^{t}\mu_{k}q_{\times }^{T}{\left(P_{\times }D_{\times }P_{\times }^{-1}\right)}^{k}k_{\text{node}}\left(v_{i},v_{i}^{\prime }\right)p_{\times }\\ =q_{\times }^{T}P_{\times }\left(\sum_{k=0}^{t}\mu_{k}D_{\times }^{K}\right)P_{\times }^{-1}p_{\times }\left(\sum_{i}^{n}\sum_{i}^{n^{\prime }}k_{\text{node}}\left(v_{i},v_{i}^{\prime }\right)\right). \end{array}$$

Equation (11) is further simplified by only taking weighted powers of a diagonal matrix. Computing the central power series here takes *O*(*n*^2^*p*) time, and the spectral decomposition is calculated as *D*_*i*_ ⊗ *D*_*j*_=*D*_×_, *P*_*i*_ ⊗ *P*_*j*_=*P*_×_, (∀*i*)*A*_*i*_=*P*_*i*_*D*_*i*_*P*_*i*_^−1^. The adjacency matrix of the investor-project interaction graph can be written as

(12) $$\begin{array}{c} A_{i}⊗A_{j}=\left(P_{i}D_{i}P_{i}^{-1}\right)⊗\left(P_{j}D_{j}P_{j}^{-1}\right)\\ =\left(P_{i}⊗P_{j}\right)\left(D_{i}⊗D_{j}\right){\left(P_{i}⊗P_{j}\right)}^{-1}. \end{array}$$

Therefore, (11) is rewritten as

(13) $$\begin{array}{c} k\left(G,G^{\prime }\right)=\left(q_{i}^{T}P_{i}⊗q_{j}^{T}P_{j}\right)\left(\sum_{k=0}^{l}\mu_{k}{\left(D_{i}⊗D_{j}\right)}^{k}\right)\left(P_{i}^{-1}p_{i}⊗P_{j}^{-1}p_{j}\right)\left(\sum_{i}^{n}\sum_{i}^{n{}^{\prime }}k_{\text{node}}\left(v_{i},v_{i}^{\prime }\right)\right). \end{array}$$

The cost of computing the two flanking factors in (15) is reduced to *O* (*n*^2^).

The article "Recommending Crowdfunding Project: A Graph Kernel-Based Link Prediction Method for Extremely Sparse Implicit Feedback" was retracted in 2023. Reasons: signs of a paper mill; suspected computer-generated content; unreliable results or conclusions; concerns about the data.

### 3.5. Graph Kernel-Based Link Predication

In this paper, the recommendation is converted into a link prediction problem. Most of the previous research works simply treat the transactions that have not happened yet as negative samples with value of 0, which introduces errors into the prediction task, for the reason behind the unhappened transaction might be the unawareness of an investor towards a project. Thus, a more suitable one-class classification algorithm is utilized in this study.

One-class SVM algorithm is implemented as the classifier [29]. The pairs of an investor and a project closer to each other have more chances to be extracted as the positive instances by this one-class classification algorithm, for it only labels the training or testing data as negative sample if it is significantly different from the positive ones. The one-class classification is calculated as the following:

(14) 12w,ξ,ρ minw2+1vl∑iξi−ρ.

We have that (*w* · *φ*(*x*_*i*_)) ≥ *ρ* − *ξ*_*i*_,  *ξ*_*i*_ ≥ 0.

The classifier function is computed as follows:

(15) $$\begin{array}{c} f\left(x\right)=\text{sign}\left(w\cdot \varphi \left(x_{i}\right)-\rho \right). \end{array}$$

The graph kernel function (*G*, *G*′)=*φ*(*G*), *φ*(*G*′)_*H*_ is provided for the one-class SVM algorithm. 〈·,·〉_*H*_ denotes a dot product in a RKHS *H*, and thus *K*(*G*, *G*′)=*φ*(*G*)^*T*^*φ*(*G*′). Euclidean distance calculation method is applied to the classification task.

Projects for each investor are ranked according to prediction scores of investor-project links to obtain the top *N* recommendations. Such prediction score for a pair (*i*, *p*) is determined as

(16) $$\begin{array}{c} f\left(\left(i,p\right)\right)=\sum_{i}a_{i}K\left(\left(i,p\right),\left(i^{\prime },p^{\prime }\right)\right)+b. \end{array}$$

Since *K*((*i*, *p*), (*i*′, *p*′))=*αk*(*G*_*i*_, *G*_*i*′_′)+*βk*(*G*_*p*_, *G*_*p*′_′), (16) can be rewritten as follows:

(17) $$\begin{array}{c} f\left(\left(i,p\right)\right)=\sum_{i}a_{i}\left(\alpha k\left(G_{i},G_{i^{\prime }}^{\prime }\right)+\beta k\left(G_{p},G_{p^{\prime }}^{\prime }\right)\right)+b. \end{array}$$

In recommendation, different projects are always compared for individual investors. Thus *a*_*i*_*αk*(*G*_*i*_, *G*_*i*′_′) remains the same for each investor in each recommendation. As shown in (17), the prediction is made based on kernel functions calculating the similarities between investors and projects, and the kernel function is determined by the features of nodes and the structures of subgraph.

The article "Recommending Crowdfunding Project: A Graph Kernel-Based Link Prediction Method for Extremely Sparse Implicit Feedback" was retracted in 2023. Reasons: signs of a paper mill; suspected computer-generated content; unreliable results or conclusions; concerns about the data.

## 4. Experiment Setup

### 4.1. Dataset Collection

The user profile on Ulule contains a list of created projects, backed projects, user's location, and user's bio; Figure 4 shows an example of a user profile. Ulule is open to anonymous users, but they only have access to ongoing campaigns and successfully funded projects and no access to failed campaigns. However, Ulule does not delete the information of any project, which means that the URL of a project is valid but cannot be retrieved by search engine once it fails to raise enough grants in the limited time of fundraising campaign. Therefore, users' choices of backing a project, namely, the investor-project pairs, are collected from the list of backed projects shown on the user profile.

Experimental dataset is built through the following procedure: (1) A list of ongoing and successfully funded projects is obtained through a Python-based web crawler to initialize the dataset; (2) information of the projects on the initial list is collected, such as project founder/founders, release date, and fundraising goal and schedule; (3) backers of the projects are collected based on the information obtained in Step 2; (4) the project list is expanded by crawling other backed projects of the collected investors obtained in Step 3 through their profile pages, including successful and failed projects, and the ongoing projects that have not reached the fundraising goals are selected; (5) Step 2–4 are repeated on the selected projects from Step 4, until all projects' information and backers' list are fully obtained; (6) other information on the collected projects is further obtained based on the former steps.

### 4.2. Dataset Description

274,292 investors with 41,894 projects that they participated in are collected from Ulule through a Python-based web crawler, in which 27,241 finished projects successfully raised enough funds, and thus the percentage of financing success rate on Ulule is approximately 65%.  Figure 5 illustrates that the number of investments of most users is less than 5, and about 82.5% of users only invest once. The total number of investor-project pairs in this dataset is 363,608, and the data sparsity is 99.98%. Therefore, the experimental dataset in this paper is extremely sparse.

As data sparsity is one of the biggest challenges for recommendation, the extant research works only include users with 5 or more transactions in experimental dataset. On the contrary, this research tests and verifies the performances of the proposed approach on datasets with different density and provides guidance for further application on choosing suitable recommendation algorithm accordingly. Therefore, the dataset is divided into three categories based on data density: extremely sparse dataset, medium sparse dataset, and less sparse dataset.

The article "Recommending Crowdfunding Project: A Graph Kernel-Based Link Prediction Method for Extremely Sparse Implicit Feedback" was retracted in 2023. Reasons: signs of a paper mill; suspected computer-generated content; unreliable results or conclusions; concerns about the data.

#### 4.2.1. Extremely Sparse Dataset

Investors with 3∼4 investments are selected from the initial dataset, and the investors with only one transaction are removed from this study. Although recommendations should be provided to the investors with only one transaction (such investors are common in reality), it is infeasible to verify the success or failure of recommendation for such investors by any algorithm if they only appear in the training data, while it is impossible to generate recommendation for them if they only appear in the testing data.

#### 4.2.2. Medium Sparse Dataset

Investors with 5∼8 investments are selected from the initial dataset, and a list of users invested in these projects is extracted.

#### 4.2.3. Less Sparse Dataset

Investors that have backed 9 or more projects are selected from the initial dataset, and a list of users invested in these projects is extracted.

Table 2 reports the descriptive statistics of the categorized datasets.

As illustrated in Table 2, the number of investors is far more than that of projects, which is similar in other public datasets, such as MovieLens, with remarkably larger number of users than that of items, since the number of users rapidly increases with numerous newcomers every year and eventually far exceeds that of products. As a result, the item-based collaborative filtering was proposed by Amazon due to the oversize user base.

### 4.3. Negative Feedback Data Collection

Most commonly used public experimental datasets for recommendation systems, such as MovieLens, contain positive and negative feedback data that shows users' “likes” and “dislikes” towards items. However, the experimental dataset collected in this paper only contains explicitly positive feedback data that shows a user's investment in projects, and the projects that the user does not invest in are not necessarily the ones that he/she dislikes; they may only be the ones that he/she is unaware of. Such data is called implicit feedback, as shown in Figure 6.

A balanced and an unbalanced collection method are applied to collect the implicit negative feedback data that are assigned “0” in Figure 6.

#### 4.3.1. Balanced Collection Method

All the projects that users does not invest in are taken as the negative feedback data, or the proportion of positive and negative feedback data is flexibly controlled according to experiment condition such as different training methods.

The article "Recommending Crowdfunding Project: A Graph Kernel-Based Link Prediction Method for Extremely Sparse Implicit Feedback" was retracted in 2023. Reasons: signs of a paper mill; suspected computer-generated content; unreliable results or conclusions; concerns about the data.

#### 4.3.2. Unbalanced Collection Method

Set a standard for negative feedback data; for example, the popular projects and the projects on top of the search result have more chances to be known to users, and thus it is highly possible that those projects that users do not invest in are due to negative sentiment (such as less interest or even dislike).

The balanced and the unbalanced collection method are applied for the extremely sparse dataset. The balanced method randomly collects 4 negative feedbacks (the projects that a user dose not invest in) for each user, and the number of users who do not invest in each project in this dataset is demonstrated in Figure 7. The result shows a uniform distribution among the 230 projects in the extremely sparse dataset.

The unbalanced method collects 4 negative feedbacks for each user according to the popularity of projects, and the distribution of the number of users who do not invest in each project in this dataset is demonstrated in Figure 8. The result shows a nonuniform distribution among the projects, and negative feedbacks are distributed mainly in 7 projects. This indicates that crowdfunding investors may not be sensitive to the popularity of projects and result in high dispersion of negative feedback data.

### 4.4. Testing and Training Dataset

The evaluation method called “Leave One Out” is utilized in this experiment, which divides a dataset containing *n* samples into two parts; the first n-1 samples are taken as training dataset, and the last 1 sample is taken as testing dataset. As a result, for positive feedback data, the projects backed by investors are sorted by transaction time, and we take the latest invested project as the testing data and the others as the training data. For negative feedback data, randomly select 99 unbacked projects for each investor as the training data and the latest unbacked project as the testing data.

### 4.5. Evaluation Metrics

The two following measures are utilized in this paper.

#### 4.5.1. Hit Ratio (HR)

To evaluate the recommending result of testing dataset,

(18) $$\begin{array}{c} HR=\frac{\text{n}}{N}, \end{array}$$

where *n* denotes the number of projects in testing dataset listed in the top-*k* recommending result and *N* denotes the total number of projects in testing dataset.

#### 4.5.2. Normalize Discount Cumulative Gain (NDCG)

Obviously, people take more interest in the top-*k* recommendation result than the bottom of the list, and the accuracy of recommendation is more about the ranking order of the top-*k* recommending list than only accurately recommending items. Therefore, set ranking weight in calculating recommendation accuracy. In other words, the error of falsely ranking a lower rank item on top of the recommending list is much bigger than that of falsely ranking a higher rank item on bottom of the list.

(19) $$\begin{array}{c} \text{DCG}=\sum_{i=1}^{10}2^{{\text{rel}}_{i}}-1/\log_{2}\left(i+1\right),\\ \text{NDCG}=\frac{\text{DCG}}{\text{IDCG}}. \end{array}$$

In the above formula, rel_*i*_ denotes the relationship of an investor and the project ranking *i*^th^ in the recommending list. As shown in (19), DCG takes the ranking order into account when calculating the recommendation accuracy by setting ranking weight 1/log_2_(*i*+1). IDCG is a normalization process, which is DCG of the perfect ranking (accurate ranking), in order to compare different recommending results. Thus, DCG∈(0, IDCG], and NDCG∈(0, 1].

The article "Recommending Crowdfunding Project: A Graph Kernel-Based Link Prediction Method for Extremely Sparse Implicit Feedback" was retracted in 2023. Reasons: signs of a paper mill; suspected computer-generated content; unreliable results or conclusions; concerns about the data.

### 4.6. Experiment Procedure

Figure 9 shows the basic experiment procedure. At first, experiment data is collected through a web crawler from Ulule and preprocessed through data cleaning and data extraction. Then, experiment dataset is divided into training dataset and testing dataset for cross-validation. After that, the training dataset is utilized to train the proposed and baseline models. Finally, the testing dataset is employed to make recommendation for each investor thereof based the trained models, and their performances are justified by comparing the recommendations with the actual investments.

As critical for inferences, node similarity, *k*_node_(·, ·), is defined based on investor/project features shown in Table 3. For example, investors from the same area tend to share similar interests, projects within the same location or category tend to have similar attractions, project description (e.g., title, blurb, and rewards) influences investors' tendency to invest and hence the success rate thereof, and almost funded projects attract more investors than less funded ones.

## 5. Experiment Results and Evaluation

### 5.1. Comparison on Datasets with Different Sparsity

Figure 10 shows the HR of datasets with different sparsity, and Figure 11 shows the NDCG of datasets with different sparsity.

Result demonstrates that the recommendation on extremely sparse dataset achieves the best performance on both evaluation metrics, the medium sparse dataset follows, and the less sparse dataset ranks the lowest. The reason may be that the graph kernel-based link prediction method performs better with larger dataset, and as Table 2 shows, the extremely sparse dataset has the largest amount of data. The extant memory-based collaborative filtering methods always suffer from data sparsity and massive data size, for similarities of users and items are hard to calculate on sparse and high-dimensional data. On the contrary, graph kernel-based method gets the user-item interaction function, which is more suitable to deal with large and sparse dataset.

The article "Recommending Crowdfunding Project: A Graph Kernel-Based Link Prediction Method for Extremely Sparse Implicit Feedback" was retracted in 2023. Reasons: signs of a paper mill; suspected computer-generated content; unreliable results or conclusions; concerns about the data.

Furthermore, crowdfunding platform such as Ulule has much sparser data than that collected in this paper, according to the statistics mentioned in section 4.2. Therefore, the proposed graph kernel-based link prediction approach should make a good performance on recommending crowdfunding projects.

### 5.2. Comparison on Different Negative Feedback Data Collection Methods

Based on the extremely sparse dataset, the recommendation performance of balanced and unbalanced negative feedback data collection methods is compared. The results are listed in Tables 4 and 5.

Tables 3 and 4 indicate that the balanced collection method performs better than the unbalanced one. This may be due to the fact that investors in the experiment dataset may not be sensitive to the popularity of projects as illustrated in Figure 11; only 7 projects are repeatedly chosen as negative feedbacks which cannot represent the other 223 projects.

### 5.3. Comparative Experiments

To evaluate recommendation performance, a ranked list of projects for each investor is generated by the proposed approach and baselines, and recommendations are compared with actual investments in the testing data.

The following are the baselines chosen to conduct the comparative experiment with the proposed approach in this paper.

#### 5.3.1. ItemPop

It is a commonly used baseline in research works on recommendation systems. It is a nonpersonalized recommendation method that ranks projects based on the popularity.

#### 5.3.2. eALS

He et al. [2] proposed a matrix factorization method based on squared loss. It takes all the unbacked projects as negative feedbacks for each user and sets weight to these negative feedbacks according to their popularity. eALS is proposed to optimize the weighted model.

#### 5.3.3. BPR

Rendle et al. [32] proposed a Bayesian-based recommendation method. Based on the partial ordering of backed and unbacked projects for each user, Bayesian analysis is applied to deduce the maximum posterior estimation, in order to optimize the ranking list.

#### 5.3.4. NIRec

Jin [33] proposed a Neighborhood-based Interaction Model for Recommendation (NIRec), which firstly analyzes the significance of learning interactions in the investor-project bipartite graph and then captures the interactive patterns between each pair of nodes through their metapath-guided neighborhoods.

The article "Recommending Crowdfunding Project: A Graph Kernel-Based Link Prediction Method for Extremely Sparse Implicit Feedback" was retracted in 2023. Reasons: signs of a paper mill; suspected computer-generated content; unreliable results or conclusions; concerns about the data.

The comparative experiments of the proposed approach in this paper and the three baselines are conducted.

Table 6 demonstrates that the proposed graph kernel-based link prediction method in this research outperforms the three baselines in both HR and NDCG. This indicates that the proposed approach performs well on extremely sparse dataset; for the data sparsity, the dataset in this paper is 99.98%.

The reason may be in the following aspects: (1) The proposed graph-based link prediction method not only computes the similarities of investors (projects) but also generates projects (investors) in the neighborhood, whereas the memory based and matrix factorization based method cannot extract enough information from neighborhood due to extreme sparsity of data. (2) On extremely sparse dataset, the local algorithms only generate locally optimal solution, whereas the proposed graph-based link prediction method generates globally optimal solution to make up for the deficiency of sparse matrix. (3) The graph kernel function computes the implicit interactions between investors and projects, which is of help to detect potential relevance of investor-project pairs, and thus generates more accurate recommendation result. (4) The neighborhood-based interaction model shares similar thoughts on recommendation with the proposed graph-based link prediction method by computing similarity based on neighborhoods in the investor-project bipartite graph but still is more complex and suffers from the smoothing effect that degrades the recommendation performance with deep layers.

## 6. Conclusion

The data sparsity of crowdfunding platforms such as Kickstarter and Ulule is over 99%, and the classic collaborative filtering algorithms have difficulty in dealing with such sparse implicit feedback. Therefore, a graph kernel-based link prediction method is proposed in this paper for personalized recommendation of crowdfunding projects. Firstly, transactions between investors and projects are obtained from Ulule through a web crawler. Secondly, the investor-project bipartite graph is established based on transaction histories. Thirdly, a random walk graph kernel is constructed and computed. Fourthly, a one-class SVM classifier is built to distinguish positive links from negative ones. Finally, top *N* recommendations are made according to the ranking of investor-project pairs.

Comparative experiments are conducted on the extremely sparse data collected from Ulule, and the results illustrate that the proposed method achieves the best performance on the extremely sparse implicit feedback compared with medium and less sparse data. The proposed method outperforms the baselines. Moreover, the balanced negative feedback collection method performs better on the extremely sparse implicit feedback than the unbalanced one.

The article "Recommending Crowdfunding Project: A Graph Kernel-Based Link Prediction Method for Extremely Sparse Implicit Feedback" was retracted in 2023. Reasons: signs of a paper mill; suspected computer-generated content; unreliable results or conclusions; concerns about the data.

Further research will be conducted in the following aspects: (1) studying other more sophisticated graph-kernel functions to better calculate the similarity of nodes and graphs; (2) exploring how to combine more node information with graph kernels, such as projects' descriptions, project categories, and user reviews; and (3) exploring how to combine different types of graph models to make recommendation and apply it to other crowdfunding platforms such as Kickstarter.

## Figures and Tables

**Figure 1:** The basic procedure of the graph kernel-based link predication method.

**Figure 2:** An example of bipartite graph.

**Figure 3:** Investor-project pairs in the bipartite graph.

**Figure 4:** An example of user profile.

**Figure 5:** The statistics of users' investments.

**Figure 6:** The user-item matrix of implicit feedback.

**Figure 7:** The distribution of negative feedbacks collected by the balanced method.

**Figure 8:** The distribution of negative feedbacks collected by the unbalanced method.

**Figure 9:** Basic experiment procedure.

**Figure 10:** HR of datasets with different sparsity.

**Figure 11:** NDCG of datasets with different sparsity.

**Table 1:** The value and the processing of nodes' features.

Category		Variable name	Variable meaning	Variable assignment	Input processing
Investor features	Numerical	investor_id	Investor ID	0∼number of investors	One-hot
		num_campaigns	Number of posted projects	Actual number	One-hot
		num_comments	Number of comments	Actual number	One-hot
		num_contributions	Number of supported projects	Actual number	One-hot
	By type	Friends	Whether to show friends	0, 1	One-hot
		E-mail	Whether to show e-mail	0, 1	One-hot
		Ins	Whether to show ins	0, 1	One-hot
		Location	Country code and state code	Actual code	One-hot

Project features	Numerical	project_id	Project ID	0∼number of projects	One-hot
		creator_campaigns	Total number of projects posted	Actual number	One-hot
		tags_num	Number of tags for the project	Actual number	One-hot
	By type	money_categories	Currency type	1∼6	One-hot
		Location	Country code and state code	Actual code	One-hot

**Table 2:** The descriptive statistics of the datasets with different sparsity.

No.	Dataset	No. of investments per user	Sparsity (%)	No. of investors	No. of projects	No. of investments
1	Less sparse dataset	9 and more	94.36	639	220	7922
2	Medium sparse dataset	5∼8	96.81	2986	229	21847
3	Extremely sparse dataset	3∼4	97.95	8598	230	40542

**Table 3:** Investor and project features.

Category	Feature	Type	Kernel
Investor	Location	Categorical	Linear
	Categories of backed/created projects	Categorical	Linear

Project	Project category	Categorical	Linear
	Project location	Categorical	Linear
	Project title	Textual	Linear
	Blurb in project description	Textual	Linear
	Reward terms	Textual	Linear
	Success or failure of fundraising campaign	Numerical	RBF
	Ongoing (funded percentage) or finished campaign	Numerical	RBF

The article "Recommending Crowdfunding Project: A Graph Kernel-Based Link Prediction Method for Extremely Sparse Implicit Feedback" was retracted in 2023. Reasons: signs of a paper mill; suspected computer-generated content; unreliable results or conclusions; concerns about the data.

**Table 4:** HR of balanced and unbalanced collection methods on extremely sparse dataset.

No. of negative feedbacks per user	Balanced method	Unbalanced method
1	0.52943	0.10329
2	0.52501	0.19405
3	0.50907	0.24883
4	0.50523	0.28936

**Table 5:** NDCG of balanced and unbalanced collection methods on extremely sparse dataset.

No. of negative feedbacks per user	Balanced method	Unbalanced method
1	0.11817	0.05372
2	0.17679	0.0856
3	0.19505	0.09459
4	0.25262	0.11475

**Table 6:** Comparison of the proposed approach and baselines on extremely sparse dataset.

Algorithms	HR	NDCG
ItemPop	0.309	0.178
eALS	0.36	0.207
BPR	0.339	0.195
NIRec	0.496	0.288
Graph kernel	0.529	0.307

## Data Availability

No data were used to support this study.
